The article "Component-Effect Relationship between HPLC Fingerprints and Lipid-Lowering Activity of Buyang Huanwu Decoction" was published in 2022. Journal: Int J Anal Chem.

# Component-Effect Relationship between HPLC Fingerprints and Lipid-Lowering Activity of Buyang Huanwu Decoction

**DOI:** 10.1155/2022/9195335

**Published:** 2022-09-26

**Authors:** Lijing Li, Kaixuan Zhou, Qiulu Zhao, Yuejie Wang, Jia Liu, Huiwei Bao

**Affiliations:** College of Pharmacy, Changchun University of Chinese Medicine, Changchun 130117, China

## Abstract

Buyang Huanwu Decoction (BHD) has lipid-lowering and antioxidant effects. In this study, HPLC was used to establish the fingerprint of extracts from different polar parts of BHD. Through the L02 cell lipid deposition model induced by oleic acid, extracts from different polar parts of BHD were administered for treatment. Oil red O staining, TG detection, and MDA detection were used to determine lipid deposition and antioxidant activity. The component-effect relationship is established by using grey relational analysis and PLSR analysis. The results showed that the extracts from different polar parts of BHD could reduce the levels of TG and MDA. The grey relational analysis showed that the peaks that contributed greatly to the reduction of TG and MDA were peaks 3, 16, 14, 10, 1, 15, 2, and 11, respectively. Peaks 1, 4, 9, 10, 14, 16, and 17 could reduce TG and MDA through PLSR analysis. According to the results of grey relational analysis and PLSR analysis, peaks 1, 10, 14, and 16 may have good lipid-lowering and antioxidant effects. This study provides a certain preliminary basis for follow-up research on lipid-lowering drugs.

## 1. Introduction

Buyang Huanwu Decoction (BHD) is a classic traditional Chinese medicine (TCM) herbal prescription that has been clinically used to treat stroke for centuries in East Asia [1]. BHD is composed of the following 7 herbs: *Radix Astragali*, *Radix Angelicae Sinensis*, *Radix Paeoniae Rubra*, *Rhizoma Ligustici Chuanxiong*, *Semen Persicae*, *Flos Carthami*, and *Pheretima* [2]. Recent studies show that BHD has a positive effect on the treatment of diabetes and atherosclerosis [3, 4]. In Chinese clinical practice, there are many cases where BHD is used in the treatment of diabetes, which greatly improves the quality of life of patients [5, 6]. Diabetic patients often show disorders of glucose and lipid metabolism. The disorder of lipid metabolism leads to the increase of triglyceride (TG) levels and lipid peroxidation in the liver, thus producing malondialdehyde (MDA), which leads to the change of cell membrane permeability and finally destroys the cell structure [7]. Clinical studies have shown that BHD can reduce patients' blood lipids and reduce a series of diseases caused by lipid metabolism disorders [8, 9]. In our previous studies, we found that BHD could reduce blood lipids and reduce lipid deposition in the liver of diabetic rats [10]. However, BHD is a complex decoction containing a variety of chemical components. Its lipid-lowering and antioxidant-active material basis are not clear, which restricts the further development of the prescription.

The article "Component-Effect Relationship between HPLC Fingerprints and Lipid-Lowering Activity of Buyang Huanwu Decoction" was published in 2022. Journal: Int J Anal Chem.

The fingerprint method provides a comprehensive characterization of the TCM components and has been used for assessing the quality of herbal medicines [11]. The component‐effect relationship is a new method that can integrate the chemical fingerprints with pharmacological effects to ensure quality and find functional constituents in TCM [12, 13]. Therefore, in this study, BHD was extracted with different polar solvents, and HPLC chromatograms of different polar parts were established to study its lipid-lowering and antioxidant effect on steatosis L02 cells. The correlation between common peaks in HPLC fingerprints and pharmacodynamic indexes was analyzed by grey relational analysis and PLSR analysis to determine the material basis of the lipid-lowering and antioxidant effects of BHD extract and to provide a preliminary basis for the follow-up research of the lipid-lowering drugs.

## 2. Research Methods

### 2.1. Materials and Reagents

Acetonitrile of HPLC grade was obtained from Fisher Scientific (Fair Lawn, NJ, USA). Buyang Huanwu Decoction was purchased from Tongren pharmacy in Jilin Province; the insects were identified by Prof. Dacheng Jiang from the Changchun University of Chinese Medicine. Gallic acid (batch number: 110831–201204) and ferulic acid (batch number: 110773–200611) were purchased from China Pharmaceutical Biological Products Verification Institute (Beijing, China). Calycosin (batch number: 20575-57-9), hydroxysafflor yellow A (batch number: 78281-02-4), and ononin (batch number: 486-62-4) were purchased from Shanghai Standard Technical Service Co., Ltd. (Shanghai, China). Z-ligustilide (batch number: G01001909024) was purchased from Chengdu Herbpurify Co., Ltd. (Chengdu, China). Kaempferol (batch number: SK8030) was purchased from Beijing Solarbio Science and Technology Co., Ltd. (Beijing, China). Oleic acid was purchased from Shanghai Aladdin Biochemical Technology Co., Ltd. (Shanghai, China). Penicillin–streptomycin solution and pancreatic enzymes were purchased from Hyclone (Logan, Utah, USA). Fetal bovine serum and RPMI 1640 Medium were purchased from Gibco (Grand Island, NY, USA). L02 cell line was purchased from Shanghai Fuheng Biotechnology Co., Ltd. (Shanghai, China). Cell counting kit-8 was purchased from Invigentech (Irvine, CA, USA). Oil red O stain kit and triglyceride assay kit were purchased from Nanjing Jiancheng Biology Engineering Institute (Nanjing, China).

The article "Component-Effect Relationship between HPLC Fingerprints and Lipid-Lowering Activity of Buyang Huanwu Decoction" was published in 2022. Journal: Int J Anal Chem.

### 2.2. Sample Preparation

The components of BHD were extracted in a heating reflux extraction system with water, petroleum ether, ethyl acetate, and n-butanol, respectively. Weigh 20 g BHD powder, add 200 mL extraction solvent, reflux extraction for 2 hours, filter and reflux again under the same conditions, and evaporate the filtrate to dry the solvent to obtain water extract, n-butanol extract, ethyl acetate extract, and petroleum ether extract, respectively. Accurately weigh an appropriate amount of B1–B4 and dissolve it with methanol to prepare a solution with a mass concentration of 75 g·L^−1^. After 0.45 *μ*m microporous membrane filtration.

### 2.3. Reference Preparation

Dissolve precisely weighed gallic acid, hydroxysafflor yellow A, ferulic acid, calycosin, ononin, kaempferol, and Z-ligustilide in methanol, and take 100 *μ*L standard samples, respectively, mixed into a reference standard solution.

### 2.4. Chromatography Conditions

Chromatographic separation was carried out on the Agilent ZORBAX SB-C18 column (250 mm × 4.6 mm, 5 *μ*m). The mobile phase consisted of 0.1% formic acid water (A) and acetonitrile (B) using a gradient elution of 1% B at 0–18 min, 1–10% B at 18–40 min, 10–15% B at 40–50 min, 15–25% B at 50–80 min, 25–50% B at 80–100 min, and 50–100% B at 100–120 min. The flow rate was 0.8 mL/min with an injection volume of 10 *μ*L, and the detection wavelength was set at 280 nm.

### 2.5. Cell Grouping and Drug Administration

The cells were divided into 6 groups: the control group (Con), the model group (Mod, medium containing 100 *μ*M oleic acid), the B1 treatment group (B1, medium containing 100 *μ*M oleic acid and 200 *μ*g/mL BHD water extract), the B2 treatment group (B2, medium containing 100 *μ*M oleic acid and 200 *μ*g/mL BHD n-butanol extract), the B3 treatment group (B3, medium containing 100 *μ*M oleic acid and 200 *μ*g/mL BHD ethyl acetate extract), the B4 treatment group (B4, medium containing 100 *μ*M oleic acid and 200 *μ*g/mL BHD petroleum ether extract).

### 2.6. Oil Red O Staining

According to the above grouping, the cells were seeded into 24-well culture plates at a density of 2 × 10^5^ cells/well. After 24 hours of cell treatment, the old medium was discarded. Add the oil red O solution for dyeing for 15 min. After dyeing, PBS was added to clean the cells 3 times, and water-based sealant was added, observed under the microscope.

### 2.7. Cell TG Assay

According to the above grouping, the cells were seeded into 6-well culture plates at a density of 8 × 10^5^ cells/well. After 24 hours of cell treatment, the old medium was discarded, and cells were collected. The TG content was detected by the TG assay kit (GPO-PAP method). The protein content was determined by the bicinchoninic acid (BCA) method. Finally, the TG content was corrected by the protein concentration per Gram; the unit of TG was mmol/gProt.

The article "Component-Effect Relationship between HPLC Fingerprints and Lipid-Lowering Activity of Buyang Huanwu Decoction" was published in 2022. Journal: Int J Anal Chem.

### 2.8. Cell MDA Assay

The cells were seeded into 6-well culture plates at a density of 8 × 10^5^ cells/well. After 24 hours of cell treatment, the old medium was discarded, and cells were collected. The MDA content was detected by the MDA assay kit (TBA method). The protein content was determined by the BCA method. Finally, the MDA content was corrected by the protein concentration per Gram, the unit of MDA was mmol/gProt.

### 2.9. Grey Relational Analysis

The grey relational analysis uses SPSSPRO online data analysis platform (https://www.spsspro.com/) for analysis. The standardized pharmacodynamic index (*X*_0_) was used as the reference sequence, and the peak area (*X*_*i*_) of the compound in the sample was used as the comparison sequence. The initial value method was used to normalize the raw data. The correlation coefficient reflects the consistency between the reference sequence and the comparison sequence. The larger the value of the correlation coefficient, the closer the comparison sequence is to the reference sequence. The correlation degree indicates the degree of similarity between each evaluation item and the reference sequence, which is calculated by the average value of the correlation coefficient. The correlation degree value is between 0 and 1. The larger the value, the stronger the correlation between the evaluation item and the reference sequence. When the correlation degree is > 0.7, it is determined that the peak has a high correlation with the drug effect [14].

### 2.10. PLSR Analysis

PLSR analysis was performed using Simca14.1 software to establish the statistical correlation between multiple dependent and independent variables. In this study, 24 chromatographic peaks were used as independent variables, while TG or MDA was used as a dependent variable to generate a regression model. The correlation between the peak areas and TG or MDA was analyzed using the PLSR model [15].

Variable importance in projection (VIP) scores indicate the contribution of independent variables to the dependent variables; high VIP scores indicate an enhanced contribution of the components to biological activities. A VIP score greater than 1 indicates that the independent variable has a marked contribution to the dependent variable [16]. The magnitude of the correlation coefficient, which indicates the degree of correlation between the phytochemical components and pharmacological activity, is directly proportional to the degree of correlation. A correlation coefficient value greater than 0 indicates that the component has a positive regulatory effect on pharmacological activity. Conversely, a correlation coefficient value of less than 0 indicates that the component has a negative regulatory effect on the activity.

The article "Component-Effect Relationship between HPLC Fingerprints and Lipid-Lowering Activity of Buyang Huanwu Decoction" was published in 2022. Journal: Int J Anal Chem.

### 2.11. Statistical Analysis

The significance test for the data obtained from the experiments performed was subjected to the one-way analysis of variance (ANOVA) using Student's *t*-tests for TG and MDA of all samples tested for BHD. The results obtained at *P* < 0.05 were interpreted as significant.

## 3. Results

### 3.1. HPLC Chromatograms of Different Polar Fractions of BHD Extracts

The HPLC chromatograms of different polar fractions of BHD extracts are shown in Figure 1. Analysis of the HPLC chromatograms of the four BHD extracts revealed variations in the phytochemical components. In total, 24 peaks were identified in all 4 extracts. The mixed reference solution is shown in Figure 2. After comparing with the reference standard, five of the 24 peaks were identified, which were gallic acid (P5), ferulic acid (P13), ononin (P16), calycosin (P18), and *Z*-ligustilide (P23).

### 3.2. BHD Inhibited Lipid Accumulation in OA-Induced Hepatocytes

Oil red O staining demonstrated that OA-induced lipid droplet accumulation in L02 cells and different polar fractions of BHD extracts inhibited the accumulation of lipid droplets (Figure 3(a)).

Different polar fractions of BHD extracts attenuated the formation of intracellular TG induced by OA, among which BHD water extract and n-butanol extract can significantly reduce intracellular TG (Figure 3(b)); the reduction rates of TG in the B1, B2, B3, and B4 groups were 51.87%, 56.97%, 46.24%, and 47.91%, respectively.

### 3.3. BHD Reduces MDA Level in L02 Cells

The MDA level in the model group was much higher than that in the normal control group. After different polar fractions of BHD extract treatment, the level of intracellular MDA decreased, among which BHD water extract and n-butanol extract can significantly reduce intracellular MDA (Figure 3(c)). The reduction rates of MDA in the B1, B2, B3, and B4 groups were 39.40%, 52.06%, 24.62%, and 30.85%, respectively.

### 3.4. Grey Relational Analysis of the Component-Effect Relationship

A grey relational analysis (GRA) was used to assess the component-effect relationship between the areas of 24 chromatographic peaks and the content of different extracts on TG and MDA. As shown in Table 1, the correlation degree of peaks 3, 16, 14, 10, 1, 5, 15, 2, and 11 with the BHD decrease TG content was higher than 0.7; the correlation degree of peaks 1, 14, 16, 3, 10, 2, 11, 13, 15, and 18 with the BHD decrease MDA content was higher than 0.7; it has a high correlation with drug efficacy.

The article "Component-Effect Relationship between HPLC Fingerprints and Lipid-Lowering Activity of Buyang Huanwu Decoction" was published in 2022. Journal: Int J Anal Chem.

### 3.5. PLSR Analysis of the Component-Effect Relationship

As shown in Figures 4(a) and 4(b), the VIP scores of peaks 4, 1, 14, 17, 24, 16, 10, 22, 9, and 23 were higher than 1, and then the correlation coefficients of peaks 4, 1, 14, 17, 16, 10, and 9 were greater than 0, this revealed that these components significantly contributed to the reduction of TG content. As shown in Figures 4(c) and 4(d), the VIP scores of peaks 4, 1, 14, 17, 24, 16, 10, 22, 9, 15, and 23 were higher than 1, and the correlation coefficients of peaks 4, 1, 14, 17, 16, 10, and 9 were greater than 0, which revealed that these components significantly contributed to the reduction of MDA content.

## 4. Discussion

One kind of herbal medicine contains dozens of natural active ingredients, while a Chinese medicine prescription is composed of several kinds of herbal medicine [14]. Therefore, identifying the active components in these complicated formulations is a significant challenge. The application of the component-effect relationship is extremely important in identifying active components in TCM preparations. Recent studies have shown that BHD has antioxidant, antiapoptotic, regulating angiogenesis, and anti-inflammatory effects [17]. In the clinical study, BHD was supplemented in patients on the basis of routine treatment. The results showed that the levels of fasting blood glucose, triglyceride, and inflammation in patients treated with BHD decreased significantly [5, 18]. However, the efficacy material basis of BHD is not clear, which restricts the development and application of prescription.

In this study, the lipid-lowering and antioxidant effects of different polar extracts of BHD were studied through cell experiments. Oil red O staining showed that OA-induced lipid deposition in L02 cells and different polar extracts of BHD had different effects on reducing lipid deposition. Then, through the detection of TG level, it has a quantitative effect on lipid deposition. The MDA level is an important index reflecting the potential antioxidant capacity of the body [19]. MDA is an end product of lipid peroxidation. It affects the mitochondrial respiratory chain complex and the key enzyme activity in mitochondria, thus intensifying cell damage. Therefore, testing the MDA level can reflect the degree of lipid peroxidation and cell damage [20]. TG and MDA were used as lipid-lowering and antioxidant indexes, respectively, and the effective components of BHD were screened by GRA and PLSR analysis. GRA and PLSR are common statistical methods to study the correlation between variables. They can predict the correlation between components and efficacy, and each has its own advantages and disadvantages. GRA is a dynamic quantitative analysis method for a development and change system. It has low requirements for sample size and data distribution law, and the correlation degree can reflect the similarity of two variable sequence geometries. PLSR provides a multilinear regression modeling method. Especially when the number of two groups of variables is large, there are multiple correlations, and the number of observational data is small, the model established by PLSR has more advantages. Therefore, through the mutual evidence and cooperation of GRA and PLSR, this paper establishes the component-effect relationship of lipid-lowering and antioxidant effects of different polar parts of BHD and obtains the material basis of pharmacodynamics.

The article "Component-Effect Relationship between HPLC Fingerprints and Lipid-Lowering Activity of Buyang Huanwu Decoction" was published in 2022. Journal: Int J Anal Chem.

The findings of this study revealed that multiple components exhibited lipid-lowering and antioxidant activities. Through the GRA, it is concluded that peaks 3, 16, 14, 10, 1, 15, 2, and 11 contribute greatly to the reduction of TG and MDA at the same time. Through the PLSR analysis, peaks 1, 4, 9, 10, 14, 16, and 17 can reduce TG and MDA at the same time. Combining the results of GRA and PLSR analysis, peaks 1, 10, 14, and 16 may have better lipid-lowering and antioxidant effects. According to the research report, peak 14 is calycosin-7-glucoside [21, 22], identified as a compound in BHD by comparing Figure 3, and peak 16 was ononin. Calycosin-7-glucoside has good antioxidant activity [23] Studies have shown that calycosin-7-glucoside may play a potential role in the treatment of type 2 diabetes [24]. Calycosin-7-glucoside and ononin in the human small intestine triggered by *β*-glucosidase-induced deglycosylation can produce calycosin and formononetin, as a result, the aglycones can be absorbed effectively into the blood circulation [25], calycosin and formononetin have been shown to be activators of peroxisome proliferator-activated receptors (PPAR*α* and PPAR-*γ*) [26]. Calycosin can reduce the level of inflammation and improve insulin resistance in high-fat-fed diabetic rats [27, 28]. Calycosin-7-glucoside can significantly ameliorate AGEs-induced HUVEC oxidative stress and apoptosis [29]. Ononin also has antioxidant activity [30], but its lipid-lowering effect is lacking in research. Formononetin can reduce lipid accumulation by activating adenosine monophosphate-activated protein kinase (AMPK) [31]. Studies have shown that the combination of calycosin-7-*β*-D-glucoside, ononin, calycosin, and formononetin in treating diabetic animals significantly improves hypertriglyceridemia [32]. In this study, peak 1 and peak 10 were not identified. Therefore, we will further identify these two unknown components and prove whether these two peaks have contributed to lipid-lowering and antioxidant activity.

The article "Component-Effect Relationship between HPLC Fingerprints and Lipid-Lowering Activity of Buyang Huanwu Decoction" was published in 2022. Journal: Int J Anal Chem.

## Figures and Tables

**Figure 1:** Chromatograms of 4 BHD extracts were captured using HPLC.

**Figure 2:** The HPLC fingerprint of the mixed reference solution.

**Figure 3:** Effect of different polar fractions of BHD extracts on oleic acid-induced steatosis in L02 cells. (a) Intracellular lipid accumulation was detected by the Oil Red O staining method using an inverted microscope (400×). (b) Intracellular TG was assayed in L02 cells. (c) Intracellular MDA was assayed in L02 cells.

**Figure 4:** PLSR analysis. (a) VIP scores predicted the TG reduction rates of 24 chromatographic peaks. (b) The coefficient of correlation of 24 chromatographic peaks with the TG reduction rates. (c) VIP scores predicted the MDA reduction rates of 24 chromatographic peaks. (d) The coefficient of correlation of 24 chromatographic peaks with the MDA reduction rates.

**Table 1:** Correlation degree of BHD extracts with their pharmacodynamics.

TG		MDA	
Peak	Correlation degree	Peak	Correlation degree

3	0.798	1	0.815
16	0.786	14	0.811
14	0.763	16	0.765
10	0.761	3	0.761
1	0.761	10	0.742
5	0.749	2	0.729
15	0.747	11	0.728
2	0.728	13	0.717
11	0.717	15	0.705
13	0.697	18	0.705
21	0.689	5	0.698
12	0.686	12	0.684
23	0.685	21	0.663
18	0.683	9	0.66
9	0.681	17	0.658
24	0.667	4	0.636
19	0.663	23	0.62
17	0.624	20	0.616
22	0.623	19	0.613
20	0.623	24	0.61
4	0.617	22	0.569
8	0.539	8	0.541
7	0.539	7	0.541
6	0.539	6	0.541

## Data Availability

The data used to support the findings of this study are available from the corresponding author upon request.
